The article "Observation of the Auxiliary Treatment Effect of Low-Frequency Nerve Therapy Instrument after Hysteroscopy for Moderate and Severe Intrauterine Adhesions Based on Intelligent Medical Treatment" was retracted in 2022. Reason: compromised peer review.

# Observation of the Auxiliary Treatment Effect of Low-Frequency Nerve Therapy Instrument after Hysteroscopy for Moderate and Severe Intrauterine Adhesions Based on Intelligent Medical Treatment

**DOI:** 10.1155/2022/2929800

**Published:** 2022-04-11

**Authors:** Mingyue Yin, Yingzheng Pan

**Affiliations:** Department of Gynecological Endocrinology, Chongqing Health Center for Women and Children, Chongqing 401147, China

## Abstract

Uterine adhesions are mainly manifested as menstrual changes in women of childbearing age and affect fertility. Resection of uterine adhesions can well restore the shape of the patient's uterine cavity and improve the patient's menstruation. However, how to promote the growth of the endometrium and prevent the recurrence of adhesions after the operation is still a major problem. This article aims to study the use of traditional treatment methods as a control and use low-frequency nerve therapy device to assist in the treatment of posterior intrauterine adhesions recurrence rate, menstrual recovery effective rate, adverse reaction rate, liver function, etc. to study the low-frequency nerve therapy device auxiliary treatment method to prevent the postoperative effect of intrauterine adhesions. This article proposes an image processing algorithm based on intelligent medical related algorithms such as deep learning, Apriori algorithm, and an improved algorithm that introduces the degree of interest and details of 140 patients diagnosed with moderate to severe intrauterine adhesions who underwent hysteroscopic TCRA surgery in a certain affiliated hospital. The medical records were followed up by hysteroscopy and electric resection, and they were randomly divided into a control group and an observation group, with 70 cases in each group. Both groups of patients were closely monitored postoperatively, followed by postoperative review, and recorded menstrual recovery and pregnancy. At the same time, we performed hysteroscopy for recurrence of endometrial adhesions. The experimental results of this article show that the actual treatment rate of the control group is 65.7%, which is much lower than the 95.7% of the experimental group. The probability of returning to normal after 3 months of menstruation in the control group was 34.0%, much lower than the 69% in the experimental group. Three months after operation, the endometrial thickness of the experimental group was much higher than that of the control group, and the RI was lower than that of the control group. The difference was statistically significant (*P* < 0.05). The clinical treatment results are satisfactory and worthy of clinical screening.

## 1. Introduction

### 1.1. Background

In recent years, with the opening of the two-child policy, the incidence and diagnosis rate of intrauterine adhesion (IUA, also known as ASherman syndrome) in my country have shown an upward development trend called the reproductive health of IUA women of childbearing age. It is one of the areas that have been seriously threatened. Patients with intrauterine adhesions often have irregular menstruation, infertility, lower abdominal pain, etc., which disturb the life and health of young IUA patients. Due to the poor tolerance of the uterus, readhesion is a higher complication after hysteroscopic uterine cavity adhesion surgery. The readhesion rate after transcervical resection of adhesion (TCRA) reaches 48%–62.5%. It not only has an impact on the treatment effect, but also has a profound impact on the patient's related life. Therefore, integrating the existing postoperative menstrual improvement is currently a factor that cannot be ignored in measuring the efficacy of hysteroscopic surgery. It is reported that, after TCRA, the menstrual recovery rate is 70%–90%. However, not all patients with IUA can get better results, especially those with high adhesions. When there is little remaining normal endometrium, it is very difficult to repair the endometrium, and the menstrual recovery rate is low, in addition to the common menstrual reduction and amenorrhea in IUA patients, lower than normal women's pregnancy rate and fertility rate that are also important factors that IUA pay attention to.

The article "Observation of the Auxiliary Treatment Effect of Low-Frequency Nerve Therapy Instrument after Hysteroscopy for Moderate and Severe Intrauterine Adhesions Based on Intelligent Medical Treatment" was retracted in 2022. Reason: compromised peer review.

### 1.2. Significance

In recent years, the pregnancy rate of patients with infertility caused by intrauterine adhesions after hysteroscopic surgery is about 50%, and the pregnancy rate of severely ill IUA women after surgery is reported to be about 30%. At the same time, in recent years, with the development of assisted reproductive technology, the vigorous development of hysteroscopy has also increased the incidence of IVF by 2.8%. However, with the continuous increase in intrauterine operations such as abortion and curettage, it has developed into a uterus after cavity adhesion, and the possibility of the patient's assisted reproductive technology failure becomes greater. Hysteroscopy in the treatment of IUA also provides a better platform for the development of reproductive infertility. Low-frequency electrical nerve stimulation is a safe, noninvasive treatment method for repairing the pelvic floor. In recent years, its scope has continued to expand. It is gradually used in the treatment of postabortion rehabilitation and endometrial thinning and has achieved certain results. Some researchers have proposed that low-frequency electrical nerve stimulation can be used to prevent uterine adhesions, but there are also some clinical studies. Therefore, this study explored the auxiliary effect of low-frequency electrical nerve stimulation on the adjuvant therapy of moderate to severe endometrial after TCRA and its influence on menstrual recovery and endometrial thickness. Therefore, integrating existing treatment methods to prevent the recurrence of postoperative adhesions is extremely important for improving the expectations of patients' fertility.

The article "Observation of the Auxiliary Treatment Effect of Low-Frequency Nerve Therapy Instrument after Hysteroscopy for Moderate and Severe Intrauterine Adhesions Based on Intelligent Medical Treatment" was retracted in 2022. Reason: compromised peer review.

### 1.3. Related Work

Hysteroscopy is a very common tool that can provide gynecologists with the ability to diagnose and treat various intrauterine diseases. The Cholkeri-Singh and Sasaki study found that this outpatient treatment provides a quick and effective relief method for women all over the world. Although hysteroscopy is simple in concept, it is related to mild and severe complications. Awareness of these difficulties and prevention and management methods are the key to achieving good surgical results. They reviewed the well-tolerated practices of hysteroscopy complications. Although the complications of diagnostic hysteroscopy and surgical hysteroscopy are rare, they can usually be prevented by thorough preoperative evaluation and appropriate intraoperative decision-making. Understanding the patient, disease, and surgical process can help the surgeon provide the patient with the best result. With proper training and education, gynecologists can safely incorporate hysteroscopy into their surgical practice [1]. However, this experimental process is not closed, so there is a certain deviation in the experimental results. To evaluate the analgesic effect of transcutaneous electrical nerve stimulation (TENS) during office hysteroscopy without sedatives, Goldstein conducted a randomized, double-blind, placebo-controlled trial. Participants were randomly assigned to active TENS, placebo TENS, or control group. Active TENS interventions include varying high frequencies (80–100 Hz), 400 microseconds, and individually adjusted high-intensity TENS applications, at levels T10–L1 and S2–S4. In the placebo group, participants were connected to the TENS unit, but without electrical stimulation. The main result is the self-reported pain intensity (0–100 mm) measured on a visual analog scale at multiple stages (entry, contact, biopsy, and residual). It has previously been reported that the smallest clinically relevant difference in visual analogue scales is 10 mm [2]. However, due to the uncertainty of the experimental process, there are still gaps in the experimental results. The purpose and background of hysteroscopic polypectomy are the gold standard for treating endometrial polyps and obtaining specimens for histological evaluation. Alberto research shows that the controversy regarding when to provide hysteroscopic polypectomy is still ongoing, especially in asymptomatic women with occasional disease. The purpose of the Alberto study was to evaluate the accuracy of hysteroscopy and Vabra sampling in diagnosing atypical hyperplasia and cancers that grow on the surface of endometrial polyps, and to study the relationship between atypical endometrial polyps and certain potential clinically associated risk factors. They evaluated 1039 hysteroscopy and identified 345 women with endometrial polyps. All patients with endometrial polyps underwent hysteroscopic polypectomy. They collected data on age, menopausal status, abnormal uterine bleeding (AUB), hormone replacement therapy, and the use of tamoxifen [3]. Although the research perspective is forward-looking, there are still many unachievable parts of the technology.

The article "Observation of the Auxiliary Treatment Effect of Low-Frequency Nerve Therapy Instrument after Hysteroscopy for Moderate and Severe Intrauterine Adhesions Based on Intelligent Medical Treatment" was retracted in 2022. Reason: compromised peer review.

### 1.4. Innovation

The innovation of this article lies in the following: (1) this article proposes an image processing algorithm based on intelligent medical related algorithms such as deep learning, Apriori algorithm, and an improved algorithm that introduces the degree of interest to provide technical support for the observation of the auxiliary treatment effect of the low-frequency nerve therapy instrument after hysteroscopy for moderate and severe intrauterine adhesions. (2) The research in this article is based on traditional treatment methods, and the low-frequency nerve therapy device is used to assist in the treatment of posterior intrauterine adhesions recurrence rate, menstrual recovery effective rate, adverse reaction rate, and liver function, as well as the curative effect of the treatment method on preventing postoperative intrauterine adhesions.

## 2. Smart Medical Related Algorithms

### 2.1. Image Processing Algorithms for Deep Learning

Due to the different angles when the images are collected, the illumination will also be different. Because the light will affect the brightness of the picture, some pictures need to be compensated for brightness in the case of large deviations in the light [4]. The progressive upsampling of image processing is shown in Figure 1.

#### 2.1.1. Brightness Compensation

Color plays a very important role in computer vision research. Color expresses the characteristics of many aspects of images. Many fields use the color characteristics of objects, such as image segmentation and target positioning [5, 6]. The color of the object will change with the intensity of the light source. The reflected image is mainly related to three factors: the color of the object itself, the reflectivity of the surface, the light source, and the characteristics of the imaging device [7]. These factors are expressed in mathematical language. Set in the RGB color model space, a point on the surface of an object in this space that is represented by *x*. The color of the point is *f*=(*R*, *G*, *B*)^*T*^. The specific mathematical expression is

(1) $$\begin{array}{c} f\left(x\right)=\int e\left(\gamma \right)s\left(x,\gamma \right)c\left(\gamma \right)\text{d}\gamma . \end{array}$$

In the formula, *e*(*γ*) represents the color distribution of the light source, *γ* represents the wavelength of the light, *s*(*x*, *γ*) represents the albedo of the object surface at point *x*, and *c*(*γ*) represents the photosensitive function of the imaging device [8, 9]. The goal of illumination estimation is to estimate the illumination *e*:

(2) $$\begin{array}{c} e=\int e\left(\gamma \right)c\left(\gamma \right)\text{d}\gamma . \end{array}$$

The article "Observation of the Auxiliary Treatment Effect of Low-Frequency Nerve Therapy Instrument after Hysteroscopy for Moderate and Severe Intrauterine Adhesions Based on Intelligent Medical Treatment" was retracted in 2022. Reason: compromised peer review.

#### 2.1.2. Grey-World Algorithm

The premise of this algorithm is that the average value of the surface reflection of all objects in the scene is without chromatic aberration, that is,

(3) $$\begin{array}{c} 1e=\frac{\int s\left(x,\gamma \right)\text{d}x}{\int \text{d}x}. \end{array}$$

*l* is a constant, and the meaning of *s*(*x*, *γ*) is the same as that of formula (1). According to this assumption and equations (1) and (2), the illumination color value can be obtained by averaging the image to obtain the following equation [10]:

(4) $$\begin{array}{c} 1e=\frac{\int f\left(x\right)\text{d}x}{\int \text{d}x}. \end{array}$$

#### 2.1.3. Max-RGB Algorithm

The condition of this algorithm is to acquire an image in a scene with white spots. The characteristic of this image is that the maximum bright color (bright color) of each RGB channel needs to be displayed in the white point at the same time [11,12]. The mathematical expression is as follows:

(5) f∞maxx,γ=1e.

*f* represents the image in this kind of scene, *e* represents the light source, and *l* is a constant. The general White Patch algorithm does not require that the above conditions must be met, and it is not required to obtain the maximum value of each RGB channel at the same point. Formula (5) can be expressed as follows:

(6) f∞maxx,γ=R∞maxx,G∞maxx,B∞maxx.

### 2.2. Apriori Algorithm

Combining the characteristics of the medical big data mining environment, this paper optimizes the Apriori algorithm by introducing the degree of interest to improve its performance [2]. The following are an analysis and comparison of the existing interest degree models:

#### 2.2.1. Probabilistic Interest Degree Model

The probability-based interest model is as follows:

(7) $$\begin{array}{c} \int \left(X⟶Y\right)=\frac{1-P\left(Y\right)}{\left(1-P\left(X\right)\right)\left(1-P\left(Y/X\right)\right)}. \end{array}$$

Among them, *P*(*X*) represents the probability of transaction *X* appearing in transaction set *D*, and the specific calculation formula is Count(*X*)/*N*; *P*(*Y*) represents the probability of transaction *Y* appearing in transaction set *D*, and the specific calculation formula is Count(*X*)/*N*; *P*(*Y*/*X*) represents the probability that transactions *X* and *Y* appear at the same time in transaction set *D*, and the specific calculation formula is Count(*X* ∪ *Y*)/*N* [13, 14].

The article "Observation of the Auxiliary Treatment Effect of Low-Frequency Nerve Therapy Instrument after Hysteroscopy for Moderate and Severe Intrauterine Adhesions Based on Intelligent Medical Treatment" was retracted in 2022. Reason: compromised peer review.

The probability-based interest degree model mainly considers the conciseness of the association rule (*X*⟶*Y*) and is affected by the support degree Supp(*X*⟶*Y*) and the subsequent item *Y* but does not consider the association rule's previous *X* to the association rule (*X*⟶*Y*) influence [15].

#### 2.2.2. Different Interest Degree Model

The difference-based interest model is as follows:

(8) $$\begin{array}{c} \int \left(X⟶Y\right)=\frac{\text{Conf}\left(X⟶Y\right)-\text{Supp}\left(Y\right)}{\max\left(\text{Conf}\left(X⟶Y\right),\text{Supp}\left(Y\right)\right)}. \end{array}$$

Among them, max(conf(*X*⟶*Y*), Supp(*Y*)) is an evaluation standard, and its function is to ensure the establishment of the condition |Int(*X*⟶*Y*| < 1. The interest degree model based on the difference will be the following item *Y*. The support degree Supp(*Y*) and the confidence degree conf(*X*⟶*Y*) are combined to reflect the probability of occurrence of the latter item *Y* under the influence of the former item *X* in the association rule (*X*⟶*Y*) [16, 17]. The greater the difference between the item *Y* support degree Supp(*Y*) and the rule (*X*⟶*Y*) confidence level conf(*X*⟶*Y*), that is, |Int(*X*⟶*Y*)| is larger, which is greater than the preset minimum interest degree threshold. When min_int, the association rule (*X*⟶*Y*), has a greater value; conversely, when |Int(*X*⟶*Y*)| is less than the minimum interest threshold min_int, the value of the association rule (*X*⟶*Y*) is smaller [18].

#### 2.2.3. Related Interest Degree Model

The interest degree model based on correlation is as follows:

(9) $$\begin{array}{c} \text{Int}\left(X⟶Y\right)=\frac{\text{Supp}\left(S\cup^{}Y\right)}{\text{Supp}\left(X\right)\text{Supp}\left(Y\right)}. \end{array}$$

Among them, Supp(*X*U*Y*)=Count(*X*U*Y*)/*N*, Supp(*X*)=Count(*X*)/*N*, Supp(*Y*)=Count(*Y*)/*N*.

#### 2.2.4. Information Volume Interest Degree Model

Based on the information volume of the interest degree model, the interest degree of the association rule (*X*⟶*Y*) is defined as

(10) $$\begin{array}{c} \text{Int}\left(X⟶Y\right)=P\left(X\right)\left[P\left(Y|X\right)\log\left(\frac{P\left(Y|X\right)}{p\left(Y\right)}\right)+\left(1-P\left(Y|X\right)\right)\log\left(\frac{1-P\left(Y|X\right)}{1-P\left(Y\right)}\right)\right]. \end{array}$$

Among them, *P*(*X*)=Count(*X*)/*N*, *P*(*Y*)=Count(*Y*)/*N*, *P*(*YX*)=Count(*XUY*)/*N* .

The article "Observation of the Auxiliary Treatment Effect of Low-Frequency Nerve Therapy Instrument after Hysteroscopy for Moderate and Severe Intrauterine Adhesions Based on Intelligent Medical Treatment" was retracted in 2022. Reason: compromised peer review.

The interest degree model based on the amount of information comprehensively considers the conciseness of the association rules (*X*⟶*Y*), the amount of information, and the similarity of the probability distributions of the preceding term *X* and the following term *Y*, and the probability of the preceding term *X* appearing *P*(*X*) is regarded as the association Rule (*X*⟶*Y*), a measure of the simplicity of the preceding item *x* [19, 20]. The more concise the association rule (*X*⟶*Y*), the fewer the occurrences of the preceding term *X*, and the higher the interest degree Int(*X*⟶*Y*) of the whole association rule (*X*⟶*Y*).

#### 2.2.5. Effect of the Interest Degree Model

The influence-based interest model is as follows:

(11) $$\begin{array}{c} \text{Int}\left(X\;⟶Y\right)=\log\frac{\text{Conf}\left(X\;⟶Y\right)/\text{Conf}\left(X\;⟶\bar{Y}\right)}{\text{Supp}\left(Y\right)/\text{Supp}\left(\bar{Y}\right)}\\ =\log\frac{N-\text{Count}\left(X\right)}{\text{Count}\left(X\right)-\text{Count}\left(X\cup Y\right)}*\frac{\text{Count}\left(X\cup Y\right)}{\text{Count}\left(Y\right)}. \end{array}$$

Among them, Con(*X*⟶*Y*) is the confidence level of the association rule (*X*⟶*Y*), $\text{conf}\left(X\;⟶\bar{Y}\right)=\left(N-\text{Count}\left(X\;UY\right)\right)/\text{Count}\left(X\right),\text{Supp}\left(Y\right)=\text{Count}\left(Y\right)/N,\text{Supp}\left(\bar{Y}\right)=\left(N-\text{ Count}\left(Y\right)\right)/N$. The influence-based interest degree model determines the association rule interest degree through the influence of the preceding item *X* on the association rule (*XY*), which can effectively measure the strong and weak association rules close to the threshold [21].

### 2.3. Introducing an Improved Algorithm of Interest

By comparing and analyzing models with different degrees of interest and actual medical data mining needs, this article proposes the following: in order to better interest models, the smart big data medical platform is divided into five parts according to its capabilities: data collection layer, data storage layer, data mining layer, enterprise-level database, and application layer [22]. Each part can form a separate sub-cloud, where the data mining layer and the application layer share the use of the data storage layer.  Figure 2 shows the development of a cloud health platform and smart medical data platform architecture.

The article "Observation of the Auxiliary Treatment Effect of Low-Frequency Nerve Therapy Instrument after Hysteroscopy for Moderate and Severe Intrauterine Adhesions Based on Intelligent Medical Treatment" was retracted in 2022. Reason: compromised peer review.

This is shown in the following equations:

(12) $$\begin{array}{c} \text{Int}\left(X\;⟶Y\right)=\text{Conf}\left(X\;⟶Y\right)-\text{Conf}\left(\bar{X}\;⟶Y\right)=\frac{P\left(X\cup Y\right)}{P\left(X\right)}-\frac{P\left(\bar{X}\cup Y\right)}{P\left(\bar{X}\right)}, \end{array}$$

(13) $$\begin{array}{c} =\frac{P\left(X\cup Y\right)-P\left(X\right)P\left(Y\right)}{P\left(X\right)\left[1-P\left(X\right)\right]}. \end{array}$$

Among them, Conf(*X*⟶*Y*) is the confidence of the association rule (*X*⟶*Y*), that is, the probability of the occurrence of the subsequent term *Y* when the preceding term *x* exists; and Conf(*X*⟶*Y*) is the confidence of the association rule (*X* > *Y*) degree, that is, the probability that the latter term *Y* appears when the former term *X* does not exist.

## 3. Auxiliary Treatment with Low-Frequency Nerve Therapy Instrument

### 3.1. Materials and Methods

#### 3.1.1. General Information

From January 2019 to October 2020, the detailed medical records of 140 patients diagnosed with moderate to severe intrauterine adhesions who underwent hysteroscopic TCRA surgery in a certain affiliated hospital were followed up. Among them, 81 had severe intrauterine adhesions and 59 had moderate intrauterine adhesions. All patients were treated with hysteroscopic electric resection and were randomly divided into control group and observation group, with 70 cases in each group. The age of the control group was 24 to 44 years old, with an average of (32.47 ± 5.2) years; the course of disease was 2–10 months, with an average of (6.18 ± 1.68) months. The observation group was 24 to 42 years old, with an average of (32.35 ± 4.26) years; the course of disease was 2–11 months, with an average of (6.59 ± 2.21) months. The general condition of the patient can be shown in Table 1.

It can be seen from Table 1 that, in this study, 127 of 140 patients with moderate to severe intrauterine adhesions and fertility requirements had a history of intrauterine surgery (90.7%), which was similar to 90% reported in the literature. Among the 140 patients, 40 had a history of abortion, 57 had a history of multiple abortions, 20 had a history of uterine curettage after missed abortion, 11 had undergone uterine cavity manipulation due to other nonpregnancy factors, and 5 had no medical abortion. Undergoing dilatation and curettage, 5 people denied any history of abortion and intrauterine surgery. There was no significant statistical difference between the control group and the observation group in terms of age, artificial abortion, missed abortion, hydatidiform moles, and other general conditions (*P* > 0.05), and each group was comparable.

The article "Observation of the Auxiliary Treatment Effect of Low-Frequency Nerve Therapy Instrument after Hysteroscopy for Moderate and Severe Intrauterine Adhesions Based on Intelligent Medical Treatment" was retracted in 2022. Reason: compromised peer review.

#### 3.1.2. Inclusion and Exclusion Criteria

Inclusion criteria: the above-mentioned diagnostic criteria for both moderate and severe IUA; have a childbirth plan, intrauterine adhesions are the only known and only infertility factor; have a history of abortion, curettage, and other uterine cavity operations, and have a history of menstrual abnormalities before surgery. In line with the principle of informed consent, patients have good compliance and receive regular follow-up visits and follow-up.

Exclusion criteria: combined with heart function level III-IV; surgical contraindications, medication allergy; diagnosis combined with other diseases that may cause abnormal vaginal bleeding, such as endometrial polyps, uterine fibroids, submucosal types, gynecological tumors, etc.; no Cooperate with the treatment plan or unwilling to complete the follow-up; excluding genital tuberculosis.

### 3.2. Research Methods

Both groups underwent TCRA surgery, and none of the patients had postoperative complications. After surgery, 3 mg/dose, 2 doses/day, for 21 consecutive days, 8 mg medroxyprogesterone acetate was added every day for 7 consecutive days from the 14th day, the two drugs were discontinued at the same time; if this is the case for discontinuation of bleeding, it should be on the fifth day of bleeding, and medroxyprogesterone acetate was added once a day for 7 consecutive days, and the drug was stopped for 3 days each time. Taking the control group as an example, the experimental group received 30 mm/sec low-frequency nerve stimulation treatment once a day and received low-frequency nerve stimulation. Acupoints: Sanyinjiao, Zhongji, Tianshu, Uterus, Guanyuan, frequency 2 Hz, current 10–20 mA, continuous 3 weeks. Three months after the operation, a TCRA hysteroscopy was performed to check for adhesions in the uterine cavity. After three months of treatment, both groups underwent hysteroscopy.

### 3.3. Observation Index and Index Evaluation Standard

Follow-up was done by telephone in March and June after the operation. The follow-up information includes the hysteroscopy of the patient at 3 months after the operation to check whether the shape of the uterine cavity is restored, as well as the effect, whether the menstruation is restored or improved or not and reissued after TCRA, the condition, frequency and degree of adhesions, postoperative complications, possible causes, pregnancy 6 months after surgery, etc. The efficacy evaluation criteria are as follows:

(1) Healing: hysteroscopy was performed 3 months after the operation, the shape and volume of the uterine cavity returned to normal, and the opening of the bilateral fallopian tubes are observed. (2) Effective: Severe uterine cavity can be restored to mild abnormality or moderate IUA. Compared with preoperatively, the adhesion area was significantly reduced, and bilateral or unilateral fallopian tube openings could be observed. (3) Invalid: No special changes in the shape of the uterine cavity. Three months after surgery, the two groups of patients were observed by hysteroscopy, the number of treatment effects was measured, and the total effective rate (total effective = treatment + effective) was measured.

The article "Observation of the Auxiliary Treatment Effect of Low-Frequency Nerve Therapy Instrument after Hysteroscopy for Moderate and Severe Intrauterine Adhesions Based on Intelligent Medical Treatment" was retracted in 2022. Reason: compromised peer review.

### 3.4. Statistical Processing

The SPSS18.0 statistical software was used for data processing, the measurement data were expressed as $\bar{X}$ ± *s*, and the *t*-test was used. The rank sum test was used for the comparison of grade data. *P* < 0.05 indicated that the difference was statistically significant.

## 4. Treatment Results and Analysis

### 4.1. Comparison of Treatment Effects between the Two Groups

In a normal menstrual cycle, the endometrium can be completely regenerated under the circulation of estrogen and progesterone. IUA is caused by various factors that cause damage to the basal layer of the patient's endometrium, the regeneration of the functional layer is stagnated, and some fibrotic hyperplasia, fibrosis, and mutual adhesions form uterine wall adhesions, which lead to the uterine cavity. A series of traumatic amenorrhea syndromes is caused by a small part or complete fit for a long time. It may be seen from previous studies that many common factors that can lead to IUA have been found, including infection and history of intrauterine and cervical canal surgery trauma, and all factors that can cause intrauterine injury or endometrial inflammation can cause IUA. The comparison of the before and after clinical treatment of moderate to severe intrauterine adhesions in the control group and the comparison of the before and after clinical treatment effects of moderate to severe intrauterine adhesions in the experimental group are shown in Figures 3 and 4, respectively.

#### 4.1.1. Comparison of Short-Term Efficacy between the Two Groups

The treatment effective rate of the control group was 65.7%, which was far lower than the 95.7% of the experimental group, and the difference was statistically significant (*P* < 0.05). The short-term efficacy comparison between the two groups is shown in Table 2.

#### 4.1.2. Comparison of Menstrual Improvement in the Two Groups after 3 Months

The clinical symptoms of IUA can cause abnormal menstrual flow (little menstruation or no menstruation at all), periodic lower abdominal discomfort with or without, recurrent or frequent miscarriage, infertility, bad pregnancy or childbirth history, etc. Menstrual abnormalities are considered to be the most typical symptoms of menstruation significantly less than before or direct amenorrhea. Secondary amenorrhea caused by IUA may be due to complete adhesions inside the cervix or complete damage to the uterine cavity. Some patients are accompanied by intermittent lower abdominal pain, which may be caused by adhesions in the cervix, resulting in unsmooth discharge of menstrual blood, which poses a serious threat to the normal health of women of gestational age. Three months after surgery, the control group had a 34.0% chance of returning to normal menstruation, which was far lower than 69% in the experimental group. The difference was statistically significant (*P* < 0.05). The comparison of menstrual improvement in the two groups at three months after surgery is shown in Table 3.

The article "Observation of the Auxiliary Treatment Effect of Low-Frequency Nerve Therapy Instrument after Hysteroscopy for Moderate and Severe Intrauterine Adhesions Based on Intelligent Medical Treatment" was retracted in 2022. Reason: compromised peer review.

#### 4.1.3. Comparison of Endometrial Thickness and RI between the Two Groups before and after Treatment

The endometrial thickness of the experimental group was much higher than that of the control group at 3 months after operation, while the RI was lower than that of the control group. The difference was statistically significant (*P* < 0.05). The RI value of the two groups at 3 months after operation was lower than that before operation. The reason may be that the thickness of the endometrium at 3 months after surgery and the thickness of the posterior membrane at 3 months after surgery are different. The reason may be that low-frequency nerve electrical stimulation can increase the excitability of muscle ovarian cells, promote new metabolism of ovarian cells, and improve ovarian blood supply, and so on. The thickness of the endometrium increased compared with that before the operation, and the difference was statistically significant (*P* < 0.05); see Table 4.

### 4.2. Comparison of Curative Effect between Patients with Moderate and Severe Intrauterine Adhesions

The comparison of the treatment effect between moderate and severe IUA patients is shown in Figure 5.

It can be seen from Figure 5 that there are statistically significant differences in the pregnancy rate of moderate IUA menstruation and severe IUA, adhesion nonrecurrence rate, and overall improvement rate (*P* < 0.05). The treatment in the experimental group can prevent recurrence, improve IUA menstrual status, increase pregnancy rate, and have a better effect on moderate intrauterine adhesions.

### 4.3. Comparison of the Number of Readhesions and the Degree of Readhesion in Severe Patients in Each Group

There was no significant difference between the number of readhesions and the degree of readhesion between the control group and the experimental group of moderate IUA patients, and there was no significant difference between the severe adhesion group (= 3.703, *P* > 0.05), as shown in Figure 6.

The article "Observation of the Auxiliary Treatment Effect of Low-Frequency Nerve Therapy Instrument after Hysteroscopy for Moderate and Severe Intrauterine Adhesions Based on Intelligent Medical Treatment" was retracted in 2022. Reason: compromised peer review.

### 4.4. Comparison of the Incidence of Adverse Reactions and Liver Function Indicators in Each Group of Patients

There was no significant difference in the incidence of adverse reactions among patients in each group (*P* > 0.05). There was no significant difference in the levels of AST and ALT in liver function among the groups (*P* > 0.05). There was no statistical difference in the level of patients in each group. See Table 5 for more information.

Hysteroscopic uterine adhesion separation surgery is very difficult. Common postoperative complications include uterine perforation, accidental trauma to the cervix, peripheral organ damage, air embolism, and uterine bleeding. In addition, patients with IUA have a history of uterine surgery, and the risk of damage to the myometrium may increase during hysteroscopy and repeated use of false tubes. Therefore, such operations should be performed by highly qualified physicians with deep experience, under the monitoring of abdominal ultrasound or laparoscopy, to avoid complications and increasing the length of the operation and reduce possible damage, reduce the risk of uterine perforation during the operation, and increase its safety. When the operation is over, it does not mean the end of the treatment process. After the operation, it is still necessary to combine treatments that effectively promote the growth of the endometrium to avoid recurrence of adhesions. The auxiliary low-frequency nerve therapy that promotes the growth of the endometrium and maintains the shape of the uterine cavity is currently the most important treatment method for preventing the recurrence of adhesions. In order to promote the growth of the endometrium, a variety of effective programs need to be coordinated. Clinicians should always seek the most appropriate and comprehensive treatment method, because a treatment method after surgery may not produce good results. There are still limitations in this study: it is retrospective study, the included sample size is small, the follow-up time is short, and the later period will be multicenter and prospective research to improve the objectivity of the research results; the mechanism of low-frequency nerve electrical stimulation to prevent intrauterine adhesions needs further study.

## 5. Conclusions

Common symptoms of intrauterine adhesions include uterine adhesions (IUA) or Asherman's sign, reduced menstruation, amenorrhea, infertility, recurrent miscarriage, and abdominal pain. In recent years, due to the increase in endometrial surgery such as abortion, the incidence of intrauterine adhesions has increased. Low-frequency nerve electrical stimulation, also known as transcutaneous acupoint electrical stimulation, is a technique derived from acupuncture therapy. It uses self-adhesive skin electrodes instead of acupuncture needles and is placed on the surface of human acupoints, mainly by stimulating uterine nerves and nerves. At the periphery, it activates the relevant uterine muscle receptors, improves the uterine microenvironment, promotes blood circulation in the endometrium and myometrium, stimulates the growth of the endometrium, increases the thickness of the endometrium, and improves the receptivity. Uterine adhesion separation is a common treatment for IUA, but it can only restore the approximate shape of the uterus. For moderate to severe IUA, the attachment recurrence rate is higher than that for mild IUA, but the pregnancy rate is lower. How to achieve nonadhesion is very important, and finding the best treatment to prevent the recurrence of endometrial adhesions is an important part of ongoing research. Uterine cavity adhesion occurs on the cervical wall, and the function of the uterine cavity destroys the basal layer of the endometrium, exposing the muscular layer tissue and causing adhesion. Hysteroscopy can determine the type, extent, nature, and degree of adhesions. In order to prevent the occurrence of IUA, the following points need to be done: (1) strengthen postoperative follow-up, pay attention to postoperative menstrual recovery, and treat recurrence as soon as possible. (2) Strengthen reproductive health education for pregnant women to avoid unintended pregnancy. Since hysteroscopy is widely used in the diagnosis and treatment of IUA, adhesions can be separated under direct vision, and the normal anatomical structure of the uterine cavity can be restored. To prevent uterine adhesions and replantation, proper dosage to promote intrauterine repair is essential. In patients with moderate to severe IUA, the endometrium is severely damaged and widely distributed. That is, the overall treatment effect of IUA severity may not be satisfactory, and clinical preventive measures should be taken to reduce adhesions.

The article "Observation of the Auxiliary Treatment Effect of Low-Frequency Nerve Therapy Instrument after Hysteroscopy for Moderate and Severe Intrauterine Adhesions Based on Intelligent Medical Treatment" was retracted in 2022. Reason: compromised peer review.

## Figures and Tables

**Figure 1:** Progressive upsampling.

**Figure 2:** Intelligent medical big data platform architecture.

**Figure 3:** Comparison of clinical treatment effects of moderate to severe intrauterine adhesions (a) Before treatment of severe intrauterine adhesions (b) After treatment of severe intrauterine adhesions.

**Figure 4:** Comparison of the effect before and after clinical treatment of moderate to severe intrauterine adhesions in the experimental group.

**Figure 5:** Comparison of the effects of patients with moderate and severe intrauterine adhesions.

**Figure 6:** Comparison of the number of readhesions and the degree of readhesion in patients with severe adhesions in each group (%).

**Table 1:** General conditions of patients.

Project	Control group	Observation group
Average age	32.47 ± 5.2 years old	32.35 ± 4.26 years old
Average number of uterine cavity operations	2.15 ± 1.5 times	2.25 ± 1.4 times
A history of abortion	20 cases (14.26%)	20 cases (14.26%)
History of multiple abortions	30 cases (21.43%)	27 cases (19.29%)
Purging the palace after a missed abortion	9 cases (6.43%)	11 cases (7.86%)
Hydatidiform mole	1 cases (0.71%)	1 cases (0.71%)
Other non-pregnancy factors uterine cavity operation	5 cases (3.57%)	6 cases (3.57%)

**Table 2:** Comparison of short-term efficacy between the two groups.

Group	Total number of cases	Cured (*n*)	Markedly effective (*m*)	Ineffective (*n*)	Total effective (*n* (%))
Test group	70	28	39	3	67 (95.7)
Control group	70	14	32	24	46 (65.7)
*X* ^2^					5.619
*P*					0.046

**Table 3:** Comparison of menstrual improvement in the two groups at 3 months after operation.

Group	Total number of cases	Normal	Increase	Constant
Test group	70	49	18	3
Control group	70	25	24	21
*Z*			6.562	
*P*			0.045	

**Table 4:** Comparison of endometrial thickness and RI between the two groups before and after treatment.

Group total	Number of cases	Observation time	Endometrial thickness (em)	RI
Test group	70	Preoperative	4.11 ± 0.61	0.72 ± 0.13
		3 months after operation	6.21 ± 0.80^∗^	0.60 ± 0.10^∗^
Control group	70	Preoperative	4.07 ± 0.57	0.74 ± 0.15
		3 months after operation	6.09 ± 0.76^∗∗^	0.67 ± 0.11^∗∗^

**Table 5:** Comparison of adverse reaction rates and liver function indexes of patients in each group.

Group	Number	Adverse reactions/*n* (%)		AST/U·L^−1^			
		Breast tenderness	Breast nodule	Dizziness and headache	Gastrointestinal reaction	Before treatment	After treatment
Test group	70	1	0	1	3	19.51 ± 4.12	18.39 ± 3.52
Control group	70	2	1	1	2	19.47 ± 44.16	18.36 ± 3.17
*X* ^2^/*F*		0.517	2.017	0.517	0.303	0.281	0.595
*P*		0.773	0.365	0.772	0.859	0.998	0.912

## Data Availability

No data were used to support this study.
